# Evolution of Novel Signal Traits in the Absence of Female Preferences in *Neoconocephalus* Katydids (Orthoptera, Tettigoniidae)

**DOI:** 10.1371/journal.pone.0012457

**Published:** 2010-08-27

**Authors:** Sarah L. Bush, Johannes Schul

**Affiliations:** Division of Biological Sciences, University of Missouri, Columbia, Missouri, United States of America; University of Exeter, United Kingdom

## Abstract

**Background Significance:**

Communication signals that function to bring together the sexes are important for maintaining reproductive isolation in many taxa. Changes in male calls are often attributed to sexual selection, in which female preferences initiate signal divergence. Natural selection can also influence signal traits if calls attract predators or parasitoids, or if calling is energetically costly. Neutral evolution is often neglected in the context of acoustic communication.

**Methodology/Principal Findings:**

We describe a signal trait that appears to have evolved in the absence of either sexual or natural selection. In the katydid genus *Neoconocephalus*, calls with a derived pattern in which pulses are grouped into pairs have evolved five times independently. We have previously shown that in three of these species, females require the double pulse pattern for call recognition, and hence the recognition system of the females is also in a derived state. Here we describe the remaining two species and find that although males produce the derived call pattern, females use the ancestral recognition mechanism in which no pulse pattern is required. Females respond equally well to the single and double pulse calls, indicating that the derived trait is selectively neutral in the context of mate recognition.

**Conclusions/Significance:**

These results suggest that 1) neutral changes in signal traits could be important in the diversification of communication systems, and 2) males rather than females may be responsible for initiating signal divergence.

## Introduction

The evolutionary origin of new characters is one of the most intriguing open questions in biology. Character origin is of particular importance in the context of communication systems, as any changes in call traits that function in mate recognition are likely to have large fitness consequences [1], [2]. These fitness consequences will be especially important for call traits that maintain reproductive isolation and hence may be involved in speciation [3], [4]. Given the great diversity among calls of closely related species of frogs and insects, the processes by which such traits diversify remain a compelling problem [5], [6].

Many hypotheses for signal evolution postulate that new call traits arise and are stabilized through female preferences, either as a result of coevolutionary processes involving the male call and female preference [7]–[9], or through receiver biases in the sensory system of females [10], [11]. According to these hypotheses, sexual selection is the mechanism of diversification and females are the initiators of change [8], [9]. How females initiate change is unclear, however, given that signal parameters responsible for reproductive isolation are often under stabilizing selection [12], [13]. Nevertheless, one prediction arising from sexual selection models is that a derived call trait should be associated with a preference for the trait by conspecific females.

Strong natural selection pressure may also force a shift in signal characters. Eavesdropping by acoustically orienting predators or parasitoids could select for call traits that reduce the localizability of the caller to unintended recipients [14]–[16]. Alternatively, if signal production is energetically costly, natural selection may favor call variations that improve energetic efficiency. We describe here a communication system that has diversified despite the apparent absence of either sexual or natural selection pressure favoring the new call trait.

Katydids of the genus *Neoconocephalus* produce simple pulsed calls that vary among species in temporal characteristics including pulse rate, pulse pattern, and presence or absence of verse structure [17]. Closely related species typically attend to different temporal characteristics for call recognition [18]–[21]. Of the 24 species with described calls, nineteen produce single pulse calls in which the pulses are evenly spaced and of equal amplitude, and five produce double pulse calls in which pulses occur in pairs with alternating pulse periods [17], [22], [23]. The pairs are generated by alternating long and short pulses, long and short intervals, high and low amplitude, or a combination of these pairings (see Fig. 1A). The phylogenetic relationship of this genus has recently been reconstructed (Fig. 1B) [24]. Phylogenetic character state reconstruction indicates that the double pulse pattern evolved five times independently from the ancestral single pulse pattern (Fig. 1B, [25]).

**Figure 1:** Double pulse pattern in the calls of *Neoconocephalus*. A. Oscillograms of calls of a single pulse species (*N. robustus*, top) and two species with double pulse pattern (*N. retusus*, *N. maxillosus*). The filled arrowheads indicate the sound produced during closing movements, open arrowheads the sound generated during the opening movements of the forewings [22]. The small opening pulses play little if any role during communication and are included as part of the silent interval between pulses [18], [19]. sp = single pulse; dp = double pulse. B Total evidence tree of *Neoconocephalus* based on AFLP, nuclear, and mitochondrial data [25]. All nodes within *Neoconocephalus* have posterior probabilities of 0.98 or above. Names of species with double pulsed calls shown in bold; arrows indicate species tested here. [Outgroups: *Belocephalus davisi* Rhen and Hebard 1916 and *Bucrates malivolans* (Scudder 1878)].

Female call recognition has been studied previously in species with the ancestral single pulse pattern as well as in three species with the novel double pulse pattern [18]–[21]. In single pulsed species such as *N. robustus* and *N. nebrascensis*, females respond to any call in which the duration of silent intervals between pulses is sufficiently short (typically 2–4 ms); remarkably, no amplitude modulation is necessary to elicit a response, provided the signal lacks long silent gaps; females respond to a continuous sine wave if the frequency matches the carrier frequency of the call [18], [19], [26]. This preference for continuous calls is the presumed ancestral recognition mechanism in the genus.

In contrast, prior work on three of the five double pulse species indicates that females require this derived pulse pattern to recognize the male call: in all three species (*N. affinis, N. bivocatus, N. triops*) females evaluate the rate of the double pulses [18], [20], [21]. Hence, in these three species, both male call and female preference are in a derived state.

Here we describe the female call recognition and selectivity of the remaining two species with double pulse calls, *N. retusus* (Scudder 1878) and *N. maxillosus* (Fabricius 1775) [17], [23], [27]. Our data indicate that although the male call is in a derived state, females use the ancestral recognition mechanism to identify conspecific males. These results are surprising because unlike existing models of the evolution of communication systems, they imply that males, rather than females, may lead the divergence in signal traits.

## Materials and Methods

We collected adult male *Neoconocephalus retusus* (Scudder 1878) and female nymphs in Boone County, Missouri (USA). *N. maxillosus* (Fabricius 1775) were raised from eggs obtained from adults collected near the towns of Luquillo and Florida in Puerto Rico. Species were identified according to [23]. Insects were maintained in the laboratory on a diet of wheat seedlings, apples, and cricket food at 20–25°C and a light/dark cycle of 14/10 hours. Following the final molt, females were given two weeks to attain reproductive condition before use in experiments.

### Call recordings for verifying the double pulse pattern

We recorded males in a temperature regulated anechoic chamber at an ambient temperature of 20±2°C (*N. retusus*) or 25±2°C (*N. maxillosus*). Males were placed individually in screen cages (15 cm diameter). Calls were recorded with a 1/4″ free field microphone (G.R.A.S. 40 BF) placed 20 cm dorsal of the calling male, amplified (G.R.A.S. 26 AC & 12 AA), high-pass filtered (1000 Hz, Krohn Hite 3202), and digitized using a custom made A/D-converter system (16 bit resolution, 250 kHz sampling rate). For temporal call analysis, we also recorded male calls with ¼″ electret microphones (RadioShack 33–3028, frequency response 30 to 18,000 Hz) attached to each cage. We recorded and analyzed a minimum of 200 pulses per male. The temporal call structure was analyzed using custom-made software with a temporal resolution of 0.1 ms. To measure the duration of pulses and intervals, we used only high quality recordings in which we could identify the pulse beginnings and endings with high accuracy. To measure the pulse periods, we marked pulse beginnings at a relative amplitude of 50%. As this measurement was much more tolerant to noise, we have larger sample sizes for the period measurements (N = 28 *N. retusus* and 13 *N. maxillosus*; Fig. 2C,D) than for the duration measurements (N = 10 *N. retusus* and 11 *N. maxillosus*; Fig. 2 A,B).

**Figure 2:** The presence of alternating pulse periods in calls of *N. retusus* and *N. maxillosus*. A, B. Mean (±95% CI) durations of alternating closing pulses and the following intervals making up pulse pairs in the calls of *N. retusus* (A, N = 10) and *N. maxillosus* (B, N = 11). The duration of the intervals includes the opening pulses (see Fig. 1A). Time bars are 5 ms. C. The ratio of the longer and shorter of the two alternating pulse periods of *N. retusus* (RET, N = 28), *N. maxillosus* (MAX, N = 13), and a species with single pulse calls (*N. robustus*, ROB, N = 13). D. The CV ratio (see methods) of the pulse periods in the calls of *N. retusus* (RET, N = 28), *N. maxillosus* (MAX, N = 13), and a species with single pulse calls (*N. robustus*, ROB, N = 13). Values close to 1 indicate that the two alternating pulse periods are from the same population, while larger values indicate that they are from different populations. The box and whisker plots in C and D denote median (bar), 25th, 75th (box), 5th, 95th (whiskers) percentile, and the mean (diamond).

To verify the double pulse pattern in the calls of *N. maxillosus* and *N. retusus* we quantified two measures: first, we measured the mean duration of the alternating pulse periods in the calls (p1 and p2 in Fig. 1A) and calculated the ratio of longer period/shorter period (i.e. p2/p1, Fig. 1). Second, we compared the coefficients of variation (CV) of p1 and p2 to that of the pooled pulse periods (i.e. the mean of both p1 and p2), by calculating the CV ratio as CV_pooled_/((CV_p1_+CV_p2_)/2). If p1 and p2 are from the same population (i.e. if the call has a single pulse pattern), then CV_pooled_ should be similar to CV_p1_ and CV_p2_ and the CV-ratio should be close to 1. If p1 and p2 are from different populations (i.e. the calls have double pulse pattern) the CV_pooled_ should be larger than CV_p1_ and CV_p2_ and the CV ratio >1. To illustrate the differences between the double pulse pattern of the two focal species and the ancestral single pulse pattern, we compare the data from *N. ensiger* and *N. maxillosus* to that of a species with single pulse pattern (*N. robustus*). Males of this species were collected in Boone County (Missouri, USA); sound recordings and analysis was conducted as in the two focal species.

### Phonotaxis (experiments 1–3)

We conducted behavioral tests on a spherical walking compensator in an anechoic chamber at 20±1°C (*N. retusus*) or 25±1°C (*N. maxillosus*). In short, the insects were placed on top of a sphere, free to walk but kept in place by compensatory sphere rotations, while acoustic signals were presented from loudspeakers located in the insect's horizontal plane. The intended direction and speed of the animal were read out from the control circuitry. The experiments were performed in the dark except for an infrared light used to monitor the movements of the animal on the sphere. For details see [18]. Experiments 1 and 2 were performed in a single season with *N. maxillosus*; experiments 1–3 were performed in a single season with *N. retusus*, and experiment 3 was repeated the following year to confirm the results. Data from both years are included below. Sample sizes ranged from 6 to 10 females per experiment and are indicated in the Results. Except for experiment 1 in *N. retusus*, all experiments were conducted in a repeated measures design.

### Stimulation (experiments 1–3)

Synthetic stimuli were generated using a custom-developed DA-converter/amplifier system (16 bit resolution, 250 kHz sampling rate). Signal amplitude was adjusted using a computer controlled attenuator and delivered via one of two loudspeakers (Motorola KSN1218C) mounted at a distance of 150 cm in the horizontal plane of the insect and separated by an angle of 115°. We measured signal amplitude using a ¼″ condenser microphone (G.R.A.S. 40BF) positioned 1 cm above the top of the sphere, and a Bruel and Kjaer (Naerum, Denmark) sound level meter (B&K 2231). All stimuli were presented at 80 dB peak SPL (re 20 µPa).

The amplitude spectra of *N. retusus* and *N. maxillosus* calls had highest amplitudes in a narrowband low-frequency component centered around 15 kHz and 11 kHz, respectively, and the frequency components at ultrasonic frequencies were at least 20 dB softer than the low frequency band in the averaged spectra [28]. To generate our stimuli, we used sinusoids of 15 or 11 kHz as carrier signal to which we subsequently applied amplitude modulations. In preliminary experiments, we identified an artificial stimulus for each species that resembled the temporal structure of the natural call and was as attractive as high quality recordings of natural calls, i.e. females responded with similar walking speed and accuracy of orientation to the synthetic stimulus and to natural calls. This artificial stimulus ( = standard call model) was used as control stimulus (see below). The call model for *N. retusus* consisted of a continuously repeated train of paired pulses, each consisting of two pulses of 3.5 ms duration with an interval of 3.1 ms in between. These paired pulses were repeated after an interval of 3.8 ms. The call model for *N. maxillosus* also consisted of a continuously repeated train of paired pulses, with pulse durations of 1.5 ms and 2.5 ms with an interval of 1.5 ms in between. These paired pulses were repeated after an interval of 1.5 ms. All pulses used in this study had rise and fall times of 0.5 ms, which are included in the pulse duration. The durations of pulses and intervals used in the experiments are therefore not directly comparable to the call measurements given in Fig. 1A, which mark pulse beginning and end at 30% relative amplitude.

For ease of reading, descriptions of stimulus manipulations are provided in the Results section.

### Experimental protocol and data analysis (experiments 1–3)

The experimental protocol is described fully in [29] and [30]. Briefly, each stimulus was presented for approximately 3 minutes. After 1.5 minutes, we switched to the second loudspeaker position and pooled the responses for analysis, eliminating any potential directional biases of individual insects. Each insect was initially presented with the control stimulus, followed by two test stimuli, then the control, etc., until all stimuli in the series were presented. We imposed a one-minute period of silence between each stimulus presentation. Individual females were typically presented with 4–7 test stimuli and 3–4 controls per series, and the sequence of test stimuli was varied among females.

We quantified female responses to the test stimuli relative to their responses to the control stimulus as a “phonotaxis score,” which represents the attractiveness of the stimulus [29]. This score incorporates three criteria that positive phonotaxis should meet: (1) walking speed to the experimental stimulus relative to the control, (2) orientation ( = relative vector length), which quantifies the extent of meandering to the experimental stimulus relative to the control, and (3) and the cosine of the angular deviation of the mean walking direction toward the experimental stimulus relative to the control. The three measurements are multiplied to generate the phonotaxis score. Scores range from approximately +1 (indicating perfect phonotaxis) to −1 (perfect negative phonotaxis), with 0 indicating no response. We present phonotaxis scores as mean and 95% confidence intervals.

## Results

### Call analysis

The analysis of male calls revealed that the calls of both species possessed alternating pulse periods (Fig. 1A). In *N. retusus* (Fig. 2A), pulses were similar in length but the silent intervals between pulses differed. In *N. maxillosus*, the two pulse periods differed primarily in the pulse duration (Fig. 2B). The ratio of longer pulse period to shorter pulse period (Fig. 2C) was 1.14±0.04 (mean ± SD, n = 28) in *N. retusus* and 1.26±0.07 (n = 13) in *N. maxillosus*. The mean ratios of both species were significantly larger than that of *N. robustus* (1.03±0.02, n = 13) a species with single pulse pattern (T-test, *N. retusus*: T = −11.3, p<0.0001; *N. maxillosus*, T = −11, P<0.0001). Similarly, the CV-ratio was much larger than 1 in both *N. retusus* (3.3±1.5 mean ± SD, n = 28) and *N. maxillosus* (4.2±1.7, n = 13), indicating that the two alternating pulse periods stem from different populations. The CV-ratios of both species were significantly larger (T-test, *N. retusus*: T = −8.49, p<0.0001; *N. maxillosus*, T = −6.74, P<0.0001) than those of *N. robustus* (mean = 1.00±0.038), n = 13. Thus, calls of both *N. maxillosus* and *N. retusus* have a double pulse pattern and differ qualitatively from the single pulse calls of *N. robustus*.

### Experiment 1

Previous studies using the same setup and protocol have shown that the single pulse species *N. robustus and N. nebrascensis* respond to unmodulated signals [18], [19], but three double pulse species do not [18], [20], [21]. To determine whether females of *N. retusus* and *N. maxillosus* require the conspecific pulse pattern for call recognition, we compared the attractiveness of an unmodulated signal (i.e. a continuous sine wave) to that of the standard call models. In both *N. retusus* and *N. maxillosus*, phonotaxis scores in response to the unmodulated signal were comparable to those for the conspecific call model (*N. retusus*: 0.72±0.25 and 0.75±0.1, n = 7; *N. maxillosus*: 0.89±0.06 and 0.88±0.19, n = 6; Fig. 3A). Statistical tests revealed no differences between the responses to the call model and the unmodulated signals (*N. retusus*: Mann-Whitney u-test, n = 7, m = 10, U = 33, p>0.5; *N. maxillosus*: Wilcoxon test, n = 7, T = 8, p>0.5). These responses resemble those obtained in species with single pulse pattern (e.g. *N. robustus*) but differ from other species with double pulse pattern (e.g. *N. bivocatus*, Fig. 3B, data from [18]), where the unmodulated signal was significantly less attractive [18], [20], [21].

**Figure 3:** Importance of the pulse structure for female call recognition. A. Phonotaxis scores (mean ± 95% CI) in response to conspecific call models (open bars) and unmodulated sine waves (black bars) in *N. retusus* and *N. maxillosus*. B. Previously published data [18] for sibling species *N. robustus* (single pulse species) and *N. bivocatus* (double pulse species) for comparison.

### Experiment 2

Next, we tested the importance of the duration of the silent intervals between pulses. Previous studies using the same setup and protocol with single pulse species have shown that the attractiveness of signals decreases as interval duration increases [18], [19]. For the experiments described here, all stimuli were comprised of a single pulse pattern. In *N. retusus*, we ran three series with pulse durations of 1, 3.5, and 14 ms; interval durations varied from 0.5 to 14 ms. Responses dropped to near zero if the interval duration was more than 5 ms (at 3.5 ms pulse duration) or 7 ms (at 1 and 14 ms pulse duration) (Fig. 4A). In *N. maxillosus*. we ran two series with pulse durations of 2.5 and 6 ms, and interval durations ranging from 1 to 3 ms. Interval durations of 2.5 ms and longer rendered the stimuli unattractive at both pulse durations tested (Fig. 4B).

**Figure 4:** Importance of interval duration on female phonotaxis. In N. *retusus* (A), interval durations were varied for three different pulse durations (1, 3.5, and 14 ms); in *N. maxillosus* (B) two different pulse durations (2.5 and 6 ms) were tested. Each point represents the mean phonotaxis scores (±95% CI) of 7–8 (*N. retusus*) or 5 (*N. maxillosus*) females.

### Experiment 3

We next tested how the degree of expression of the double pulse pattern affected the attractiveness of the calls. Due to difficulties raising and maintaining the tropical *N. maxillosus* in the laboratory, we restricted this experiment to *N. retusus*. We generated a series of stimuli that had identical numbers of 3.5 ms pulses per time, with pulse patterns that varied from single pulse to double pulse patterns by moving every other pulse closer to the preceding pulse. The ratio of the two pulse periods ranged from 1 ( = single pulse pattern) to above 2 ( = extreme double pulse). The population mean of male calls was a ratio of 1.13±0.05 (n = 39) (Fig. 5 B).

**Figure 5:** Absence of female preference for the double pulse structure. Top: Phonotaxis scores (mean ± 95% CI) of *N. retusus* females toward calls that vary from single pulses to extreme double pulses as measured by the ratio of period 2/period 1 (p2/p1, see inset). The experiment was run in two consecutive years with different females. N = 9 (year 1) and N = 10 (year 2). Bottom: histogram of the ratio of long to short pulse period (p2/p1) in a population of male *N. retusus* calls (n = 39).

We performed this experiment with 9 females (Fig. 5 A, year 1) and found that the single pulse pattern was as attractive as a double pulse pattern with a ratio of pulse periods (1.15) similar to the population mean. In the complete range tested, the ratio of pulse periods did not influence female responses significantly (repeated measure ANOVA, F_3,5_ = 1.0567, p = 0.45). Because we were surprised that females had no preference for this call parameter, we repeated the experiment the following year using a narrower range of stimuli and 10 new females (Fig. 5 A, year 2). Again female responses were high in the complete stimulus range tested; statistical analysis failed to detect any influence of the ratio of pulse periods (repeated measure ANOVA, F_4,5_ = 0.4163, p = 0.79). Thus in both years we found that the presence or absence of the double pulse pattern had no effect on the attractiveness of the signal and hence does not influence the reproductive fitness of males.

## Discussion

We studied female call recognition and preferences in two *Neoconocephalus* species with a derived pulse pattern in male calls. Females evaluated the duration of the silent intervals between the pulses and responded when these intervals were short enough. Surprisingly, females of *N. retusus* responded equally well to call models with the ancestral single pulse pattern as to calls with the conspecific double pulse pattern.

Katydids generate sound by opening and closing their forewings. The opening movements produce low amplitude 'opening pulses,' which are typically irrelevant for female phonotaxis and are often omitted from call descriptions. The closing movements produce loud pulses. In species with the ancestral single pulse pattern, the forewings are opened and closed with a uniform rate [22], [31]. Double pulses are produced by a distinct motor pattern in which the wings are opened fully, closed part way (generating the first pulse of the pair), opened fully again, and then closed fully (generating the second pulse) ([22], [31]. The resulting call is characterized by two alternating pulse periods. This pattern is qualitatively different from the ancestral single pulse call (Fig. 2), as it is caused by a distinctly different motor pattern and it introduces an additional temporal parameter to the calls, i.e. the rate of pulse pairs. Thus, our data concern the origin of a qualitatively new call trait, rather than the quantitative differences (e.g., in chirp rate or fundamental frequency) that characterize many other studies of acoustic communication in insects and anurans [12], [32], [33]. Double pulses occur in the call of several genera of Tettigoniids [31], crickets [34], and in the flashpatterns of fireflies [35].

In several Tettigoniid groups, the double pulse pattern is a critical part of the species isolation mechanism. In three *Neoconocephalus* species with double pulse calls female call recognition relies heavily on this call parameter [18], [20], [21]. In one of them (*N. bivocatus*) and in *Tettigonia viridissima*, the double pulse pattern is the sole feature used by females to distinguish between conspecifics and males of sympatric sibling species [18], [29]. The present study may thus contribute to our understanding of reproductive isolation and hence speciation in this group.

### Female call recognition is in the ancestral state

The results of all three experiments indicate that although the males of *N. retusus* and *N. maxillosus* produce double pulse calls, the female recognition mechanism is typical of species with single pulse calls. In the single pulse species *N. robustus* and *N. nebrascensis*, female call recognition is limited by the duration of gaps between pulses, with maximum tolerated gaps comparable to those we found here [18], [19]. Moreover, as in *N. retusus* and *N. maxillosus*, females of the single pulse species are attracted to signals without amplitude modulation [18], [19], [26]. Thus, whereas the male calls of *N. retusus* and *N. maxillosus* are in a derived state, the female recognition mechanism remains in the presumed ancestral state typical of species with single pulse calls.

The ancestral recognition mechanism of *N. retusus* and *N. maxillosus* contrasts sharply with the derived mechanisms found in the other three species with double pulse calls (*N. affinis, N. bivocatus*, and *N. triops*). Although each species utilizes a different recognition mechanism, females of all three species exhibit a strong preference for the derived pattern: they respond only when the double pulse rate is close to that of the conspecific call [18], [20], [21]. Note that in *N. retusus* and *N. maxillosus*, strong responses occurred at dramatically varying rates: in *N. retusus* stimuli with rates of 143 Hz (3.5 ms pulse, 3.5 ms interval) and 58 Hz (14 ms pulse, 3.5 ms interval) were highly attractive; *N. maxillosus* responded strongly to pulse rates of 285 Hz (2.5 ms pulse/1 ms interval) and 143 Hz (6 ms pulse 1 ms interval). The lack of attention to pulse rate provides further evidence that *N. maxillosus* and *N. retusus* use the recognition system typical of single pulse species rather than that of double pulse species.

### Do sexual or natural selection drive the evolution of the double pulse pattern?

The results of the final experiment (Fig. 5) demonstrated that female *N. retusus* had no preference for either the derived double pulse pattern or the ancestral single pulse pattern. Female *N. maxillosus* are also unlikely to prefer the double pulse over the single pulse pattern, as the shorter intervals found in single pulse calls render the calls more attractive, if anything (Fig. 4). The absence of a preference for the derived call pattern supports the hypothesis that female choice did not drive the evolution of the double pulse pattern in *N. retusus* and *N. maxillosus*. Sexual selection could nevertheless influence call pattern if the double pulse call is more easily localized by females or if it is used in intrasexual interactions among males. Neither explanation is supported. The calculation of the phonotaxis score incorporates both attractiveness and localizability; poorly localized signals result in low vector length and consequently low phonotaxis scores. Female scores were high to single pulse calls, double pulse calls, and calls without amplitude modulation. The double pulse call also plays no role in competitive or territorial interactions among males. Call interactions among male *Neoconocephalus* occur only at the level of chirps or verses [36], [37] but not at the level of pulses [38].

The transmission of sound in the field may also provide selection on male calls, as temporal patterns may become distorted due to reflections [39]. Given that unmodulated signals are as attractive as the conspecific pattern (Fig. 3), degradation of the pattern during transmission does not affect attractiveness in these species. Thus, sound transmission does not provide an explanation for the evolution of double pulses in *N. retusus* and *N. maxillosus*.

In the absence of sexual selection pressure, is it possible that natural selection has driven the evolution of the double pulse call? Natural selection could alter call parameters either through enhanced energy efficiency of call production, through reduced attraction of acoustically orienting parasitoids [14]–[16], or through interspecific interference [40]. These explanations are unlikely in this system. The double pulse call requires the same number of wing movements as the single pulse call; only the spacing of the pulses is altered. If there were selection to save energy during calling, males of both *N. retusus* and *N. maxillosus* could have reduced their pulse rates further if they had maintained the single pulse pattern; the switch to double pulses introduces longer gaps, which lower the attractiveness of the signals and impose a higher minimum pulse rate. Finally, pulse rates in *Neoconocephalus* vary tremendously (12–300 Hz) among both single and double pulse species [17]. The majority of species call at the higher pulse rates, suggesting that energetic constraints on pulse rate have not been a driving force on call evolution in this genus.

Acoustically orienting parasitoids may profoundly influence the evolution of acoustic signaling [14]–[16]. New world katydids (including *Neoconocephalus*) are the host of tachinid flies [41]. Double pulses do not appear to provide protection from the fly, given that 70–90% of males may be parasitized both in single pulse (*N. robustus*) and double pulse species (*N. triops*) [41]. *N. maxillosus* in Puerto Rico (*unpublished*), and *N. retusus* in Florida were also heavily infested, and large numbers of flies can be trapped by broadcasting the *N. retusus* call [42]. Finally, there is no obvious reason to assume that signals with double pulse pattern would be more difficult for a predator to localize than a signal with single pulse pattern.

Reproductive interference in the form of incomplete species recognition has been postulated to select for divergent male calls in a variety of other taxa [40], but is unlikely to explain the pattern we describe here. Any syntopic congeners in which females use the ancestral recognition mechanism could indeed have been attracted to the (ancestral) single pulse call of *N. retusus* or *N. maxillosus*. A shift from single to double pulses does not prevent this occurrence, however, as is demonstrated by the results shown here; heterospecific females with the ancestral recognition mechanism would not be expected to distinguish single from double pulse calls any more effectively than do female *N. retusus*. It should also be noted that the lack of external spermatophores in *Neoconocephalus* renders a low cost to males of mismatched mating relative to some other Tettigoniids.

Thus, it appears that neither sexual selection nor natural selection provide convincing explanations for the evolution of the double pulse pattern.

### If not sexual or natural selection, what then?

Double pulses have arisen five times independently in *Neoconocephalus* and contribute significantly to reproductive isolation in three of the five species through reduced attractiveness of the single pulse pattern [18], [20], [21]. Double pulses also occur in numerous other katydid genera [23], [31] suggesting that pulse pattern is a pliable trait with a propensity to evolve a double pulse structure. The lack of a female preference for either single or double pulse patterns in *N. retusus* and *N. maxillosus* implies that the change in the male call is selectively neutral; males can introduce double pulses without any effect on reproductive fitness. If double pulses arise by chance, the new trait may spread by drift through the population. If females subsequently evolve a preference for the trait, the double pulse pattern may become stabilized. Small changes in the expression of ion channels may significantly influence the temporal selectivity of neurons [43], suggesting that few mutations may account for the differences in call recognition mechanisms observed in *Neoconocephalus* and other insect and anuran systems [20], [44]. In the absence of a change in female preferences, the trait may remain in the population or it may be lost. In this respect, the current situation in *N. maxillosus* and *N. retusus* may be temporary in evolutionary time.

The ranges of *Neoconocephalus* species in North and Central America must have changed dramatically during the Pleistocene with the advancing and retreating of glaciations. As these katydids are excellent fliers, they were potentially repeatedly influenced by founder effects. Genetic drift may thus have had profound effects on the recent diversity of this group.

Genetic drift takes place in all evolving systems and hence is inherently the null-hypothesis when considering the evolution of a trait. As it is impossible to find conclusive evidence for the null hypothesis, it can only be supported by the absence of evidence for alternative hypotheses. Therefore, we cannot fully exclude the possibility that double pulses evolved due to selection; selective advantages may have existed in the past, for example, but are no longer detectable. In the absence of a convincing selective advantage, however, the neutral hypothesis provides a parsimonious explanation for the origin of double pulses in this system.

Sexual selection is undoubtedly an important mechanism of signal divergence in many systems; numerous studies have looked for and identified female preferences for exaggerated male traits [45]. Accordingly, sexual selection is typically thought to explain most of the diversity of sexual signals [9]. In contrast, neutral hypotheses for the diversification of acoustic communication systems have only rarely been considered explicitly [e.g., 32,46]. Our results indicate that genetic drift is a parsimonious and reasonable explanation in at least some systems and that it might even account for a much larger part of the diversity in signal traits than generally assumed. We propose, therefore, that neutral hypotheses should be explicitly considered when studying the evolution of communication systems.

Our data also indicate that males are able to introduce novel call traits that ultimately may be used for species recognition: given that three of the five *Neoconocephalus* with double pulses evaluate the rate of double pulses for call recognition, this pulse pattern is responsible for maintaining reproductive isolation. Thus males may initiate the divergence of communication systems which in turn can lead to reproductive isolation and speciation. We suggest that the role of males in signal divergence and in the evolution of reproductive isolation should be considered.
